# Optimal Control and Stability Analysis of an SEIR Model with Infectious Force in Latent Period

**DOI:** 10.1155/2022/7596421

**Published:** 2022-06-15

**Authors:** Li Jiayi, Li Sixian, Shi Weixuan, Hu Manfeng, Zhang Jingxiang

**Affiliations:** School of Science, Jiangnan University, Wuxi, Jiangsu 214122, China

## Abstract

In this paper, an SEWIR epidemic model with the government control rate and infectious force in latent period is proposed. The conditions to the existence and uniqueness of disease-free and endemic equilibrium points in the SEWIR model are obtained. By using the Hurwitz criterion, the locally asymptotic stability of disease-free and endemic equilibrium points is proved. We show the global asymptotic stability of the disease-free equilibrium point by the construction of Lyapunov function and LaSalle invariance principle. The globally asymptotic stability of the endemic equilibrium is verified by numerical simulation. Several optimal control strategies are proposed on controlling infectious diseases.

## 1. Introduction

Since the outbreak of COVID-19, the global economy and social stability have been severely affected. Subsequently, the control strategies of COVID-19 infection have become the focus of research. SEIR is a commonly used model in epidemiology. It splits the entire group into four compartments: susceptible ones, exposed ones, infected ones, and recovered ones. Early in the research, many researchers considered fewer factors, and most of them directly used SEIR model to study and analyze epidemic diseases. With the deepening of research, some mathematicians found that there are more factors which affect the prediction and control of epidemic diseases, and even there are coupled dynamic changes among the factors. In the process of analyzing the transmission paths and control strategies of epidemic diseases, they have constructed lots of models for different situations to formulate the optimal strategies. Almeida et al. [1] studied an SEIR epidemic model which splits the recovery rate of infected population into two categories: without and with medical treatment. The numerical change curve of the four groups was simulated under the condition of controlling the economic cost. Carcione et al. [2] investigated an SEIR epidemic model similar to the one described in [1]. They replicated the infection and death curves by altering the four populations' baseline values, the transition rate from exposure to infection, and the recovery rate of infectious population. The importance and effectiveness of isolation and medical level in stopping the spread of the virus were verified. Khan et al. [3] considered nonlinear morbidity with a saturation constant and introduced the susceptibility for recovered individuals and medical control function into the SEIR model. It can be concluded that the optimal method to control the disease is the proper use of treatment. Several studies have demonstrated that boosting the quality of medical care during an outbreak of epidemic significantly increases the rate of recovery; however, it has no effect on limiting the transmission of the infection. Considering the factors affecting the outbreak, one of the most effective and cost-efficient control strategies, such as centralized or home isolation, are frequently implemented. Auger and Moussaoui [4] studied an SEIR epidemic model with three scenarios: individual residences, workplaces, and high-density public places based on the law of population density changing with time. Simultaneous, improving immunity through vaccination can be held accountable as an effective strategy for controlling epidemic diseases. In infectious disease dynamics, there exists two categories: continuous vaccination [5–10] and pulse vaccination [11–13]. Sen et al. [5] constructed an SIR model with constant vaccination control, and a vaccination control method was proposed. In [6], the authors studied an SEIR model including asymptomatic and dead-infectious subgroups. And, feedback vaccination as well as antiviral treatment control measures was included in the model. Nistal et al. [7] presented a discrete SEIADR model by considering diseases where infected corpses are still infectious. They introduced two types of vaccination. It was indicated that susceptible populations decrease, while recoveries increase under constant vaccination. Jiao and Shen [9] studied a more general SEIR model by introducing disease transmission rate with seasonal forcing and the rate of losing immunity of recovered population. They proposed and evaluated some control strategies by adjusting the transfer rate and simulating the population change curve under different isolation measures. However, it is practically difficult to achieve universal continuous vaccination. Hence, pulse vaccination was introduced to prevent diseases by regular vaccination. The effectiveness of this preventive measure has been proved successively [11–13].

Nowadays, most countries have implemented control measures such as vaccination, medical testing, isolation of foreign populations, close contacts and subclose contacts of diagnosed cases, and medical treatment. As a general rule, the strength of the government to implement epidemic control measures are closely related to the spread and control of epidemic. To further investigate the impact of government intervention and vaccination on the transmission kinetics, we construct a government intervention model. Additionally, the model is improved based on the traditional SEIR model under the measures taken to centrally quarantine populations tested positive after regional outbreaks in China. Given that the exposed population is still infectious, if a portion of the exposed population is medically quarantined in time, it will greatly limit the infectivity of the virus. Thus, the probability of further spread of the epidemic will be reduced, thus allowing for rapid identification and disposal and cutting off the transmission chain. Based on the above, we divide the exposed parts into two compartments: unquarantined and quarantined. Also, we introduce the government control rate and construct an SEWIR epidemic disease model with vaccination and government control.

In this paper, the whole population *N*(*t*) can be split into five divisions, designated by *S*(*t*), *E*(*t*), *W*(*t*), *I*(*t*), and *R*(*t*). *S*(*t*) is the quantity of susceptible individuals who have no immunity to the COVID-19 virus. *E*(*t*) denotes the quantity of unquarantined exposed individuals. *W*(*t*) stands for the quantity of quarantined exposed individuals. *I*(*t*) denotes the quantity of infected individuals who exhibit symptoms and are capable of propagating the disease. *R*(*t*) represents the quantity of recovered individuals with normal medical test and immunity to COVID-19 virus. Furthermore, we obtain *N*(*t*) = *S*(*t*) + *E*(*t*) + *W*(*t*) + *I*(*t*) + *R*(*t*). In Figure 1, the SEWIR model's transmission mechanism is depicted.

Based on the transmission mechanism, the SEWIR epidemic model with vaccination and government control is constructed with the form:

(1) $$\begin{array}{c} \left\{\begin{array}{c} \frac{\text{d}S}{\text{d}t}=-\beta I\left(t\right)S\left(t\right)+\Lambda \left(1-m\right)+k_{2}W\left(t\right)-mS\left(t\right)-\mu S\left(t\right),\\ \frac{\text{d}E}{\text{d}t}=\beta I\left(t\right)S\left(t\right)-k_{1}E\left(t\right)-\varepsilon E\left(t\right)-\mu E\left(t\right),\\ \frac{\text{d}W}{\text{d}t}=k_{1}E\left(t\right)-\vartheta W\left(t\right)-k_{2}W\left(t\right)-\mu W\left(t\right),\\ \frac{\text{d}I}{\text{d}t}=\varepsilon E\left(t\right)-\vartheta I\left(t\right)-\gamma I\left(t\right)-\mu I\left(t\right),\\ \frac{\text{d}R}{\text{d}t}=\vartheta W\left(t\right)+\vartheta I\left(t\right)+m\left(\Lambda +S\left(t\right)\right)-\mu R\left(t\right), \end{array}\right. \end{array}$$

where *β* denotes the ratio of infected individuals infecting susceptible ones, *m* denotes the vaccination success rate of the susceptible individuals which represents the probability of getting immunity after vaccination, *ε* denotes the conversion rates from unquarantined exposed population to infected populations, *k*_1_ denotes the government control rate, *ϑ* denotes the recovery rate, *k*_2_ denotes the autoimmune virus rate, Λ denotes the population replenishment rate including foreign population and newborns, *μ* is the natural mortality, and *γ* represents the disease mortality.

The overall structure of this paper is listed as follows: Section 2 recalls some related analysis tools.  Section 3 addresses the existence and uniqueness of equilibrium points for (2).  Section 4 analyses the stability of (2) about equilibrium points.  Section 5 simulates the relevant results and analyze the impact of vaccination and government control on infectious diseases.  Section 6 proposes some optimal control strategies for infectious illnesses.

## 2. Preliminary

In this section, we briefly recall some related analysis tools. For more details, the interested reader may refer to [14–16].

**Lemma 1 (Routh–Hurwitz theorem [14]).**

Consider the characteristic equation

(2) $$\begin{array}{c} \lambda^{n}+b_{1}\lambda^{n-1}+b_{2}\lambda^{n-2}+\cdots +b_{n-1}\lambda +b_{n}=0. \end{array}$$

There exist negative real parts for all *λ* in case

(3) $$\begin{array}{c} \Phi_{k}=\left|\begin{array}{ccccc} b_{1} & b_{3} & b_{5} & \ldots & b_{2k-1}\\ 1 & b_{2} & b_{4} & \ldots & \vdots \\ 0 & b_{1} & b_{3} & \ldots & \vdots \\ 0 & 1 & b_{2} & \ldots & b_{2k-4}\\ \vdots & \vdots & \vdots & \vdots & \vdots \\ 0 & 0 & 0 & 0 & b_{k} \end{array}\right|>0. \end{array}$$

If *k* > *n*, then *b*_*k*_=0, where *k*=1,2,3,…, *n*.

**Lemma 2 (Lyapunov's stability theorem [15]).**

Let *V* be a continuous differentiable positive definite function. If it enables $\dot{V}$ to be negative semidefinite, then the origin is stable; if it enables $\dot{V}$ to be negative definite, then the origin is asymptotically stable. When the condition of asymptotic stability holds globally as well, while *V* is radially unbounded, then the global asymptotic stability of the origin can be obtained.

**Lemma 3 (LaSalle invariance principle [16]).**

Given a system $\dot{x}=f\left(x\right)$, in which *f* is continuous. Let Ω ⊂ *D* be a positive invariant tight set of the system. Let *V* : *D*⟶*R* be a continuous differentiable function and satisfy positive definiteness. *M* is defined as the largest invariant set within $E:=\left\{x|\dot{V}\left(x\right)=0\right\}$. If the system $\dot{x}=f\left(x\right)$ starts in Ω, then with *t*⟶*∞*, the system is bound to converge to *M*.

## 3. Existence and Uniqueness of Equilibrium Points

Since the equation for *R*(*t*) is independent from other equations, then the dynamics of model (1) is qualitatively equivalent to the dynamics of model given by

(4) $$\begin{array}{c} \left\{\begin{array}{c} \frac{\text{d}S}{\text{d}t}=-\beta I\left(t\right)S\left(t\right)+\Lambda \left(1-m\right)+k_{2}W\left(t\right)-mS\left(t\right)-\mu S\left(t\right),\\ \frac{\text{d}E}{\text{d}t}=\beta I\left(t\right)S\left(t\right)-k_{1}E\left(t\right)-\varepsilon E\left(t\right)-\mu E\left(t\right),\\ \frac{\text{d}W}{\text{d}t}=k_{1}E\left(t\right)-\vartheta W\left(t\right)-k_{2}W\left(t\right)-\mu W\left(t\right),\\ \frac{\text{d}I}{\text{d}t}=\varepsilon E\left(t\right)-\vartheta I\left(t\right)-\gamma I\left(t\right)-\mu I\left(t\right). \end{array}\right. \end{array}$$

The unknown *R*(*t*) can be determined correspondingly from

(5) $$\begin{array}{c} \frac{\text{d}R}{\text{d}t}=\vartheta W+\vartheta I+m\left(\Lambda +S\right)-\mu R. \end{array}$$

It follows from (4) that

(6) $$\begin{array}{c} \frac{\text{d}S}{\text{d}t}+\frac{\text{d}E}{\text{d}t}+\frac{\text{d}W}{\text{d}t}+\frac{\text{d}I}{\text{d}t}=\Lambda \left(1-m\right)-\vartheta \left(W+I\right)-\gamma I-mS-\mu \left(S+E+W+I\right)\\ \leq \Lambda \left(1-m\right)-\mu \left(S+E+W+I\right). \end{array}$$

Furthermore, we have

(7) $$\begin{array}{c} \lim\sup_{t⟶\infty }\left(S\left(t\right)+E\left(t\right)+W\left(t\right)+I\left(t\right)\right)\leq \frac{\Lambda \left(1-m\right)}{\mu }. \end{array}$$

Considering the biological significance of the model, the dynamic properties of model (2) are only discussed in the closed set Ω, which is defined by

(8) $$\begin{array}{c} \Omega =\left\{\left(S,E,W,I\right)|0\leq S+E+W+I\leq \frac{\Lambda \left(1-m\right)}{\mu },\;S\geq 0,E\geq 0,W\geq 0,I\geq 0\right\}. \end{array}$$

It can be shown that Ω is positive and invariant. Obviously, there exists a disease-free equilibrium point *P*_0_(0,0, *S*_0_, 0) ∈ *∂*Ω with *S*_0_=Λ(1 − *m*)/*m*+*μ* for model (2). Furthermore, the basic reproduction number *R*_0_ will be applied to the proof of the existence and uniqueness of equilibriums. Relevant methods are presented in [17, 18].

Let us set **x**=(*E*, *I*, *S*, *W*)^*T*^. Then, model (2) becomes

(9) $$\begin{array}{c} \frac{\text{d}x}{\text{d}t}=\Gamma \left(x\right)-\Psi \left(x\right), \end{array}$$

with

(10) $$\begin{array}{c} \Gamma \left(x\right)={\left(\beta IS\;000\right)}^{T},\\ \Psi \left(x\right)=\left(\mu +k_{1}+\varepsilon \right)E,\\ \left(\mu +\vartheta +\gamma \right)I-\varepsilon E,\\ \beta IS+\left(\mu +m\right)S-k_{2}W-\Lambda \left(1-m\right),\\ \left(\mu +\vartheta +k_{2}\right)W-k_{1}E. \end{array}$$

The Jacobian matrix of Γ(*x*) and Ψ(*x*), when evaluated at *P*_0_(0,0, *S*_0_, 0), is as follows:

(11) $$\begin{array}{c} D\Gamma \left(P_{0}\right)={\left(\begin{array}{cc} F_{2\times 2} & O_{2\times 2}\\ O_{2\times 2} & O_{2\times 2} \end{array}\right)}_{4\times 4},\\ D\Psi \left(P_{0}\right)=\left(\begin{array}{cccc} \mu +k_{1}+\varepsilon & 0 & 0 & 0\\ -\varepsilon & \mu +\vartheta +\gamma & 0 & 0\\ 0 & \beta S_{0} & \mu +m & -k_{2}\\ -k_{1} & 0 & 0 & \mu +\vartheta +k_{2} \end{array}\right), \end{array}$$

where *O*_2×2_ denotes second-order zero matrix and $F_{2\times 2}=\left(\begin{array}{cc} 0 & \beta S_{0}\\ 0 & 0 \end{array}\right)$.

Let

(12) $$\begin{array}{c} V_{2\times 2}=\left(\begin{array}{cc} \mu +k_{1}+\varepsilon & \text{0}\\ -\varepsilon & \mu +\vartheta +\gamma \end{array}\right). \end{array}$$

Consequently, the basic reproduction number is

(13) $$\begin{array}{c} R_{0}=\rho \left(FV^{-1}\right)=\frac{\beta \varepsilon S_{0}}{\left(\mu +k_{1}+\varepsilon \right)\left(\mu +\vartheta +\gamma \right)}. \end{array}$$

**Theorem 1 .**

If *R*_0_ > 1, model (2) has *P*_0_(0,0, *S*_0_, 0) and endemic equilibrium point *P*^*∗*^(*E*^*∗*^, *I*^*∗*^, *S*^*∗*^, *W*^*∗*^). Otherwise, there exists only *P*_0_(0,0, *S*_0_, 0), where *S*_0_=(Λ(1 − *m*)/*m*+*μ*), *S*^*∗*^=(*T*_1_*T*_2_/*βε*), *E*^*∗*^=*T*_3_*T*_1_*T*_2_*θ*(1 − *R*_0_)/*βε*(*k*_1_*k*_2_ − *T*_1_*T*_3_), *I*^*∗*^=(*ε*/*T*_2_)*E*^*∗*^, *W*^*∗*^=(*k*_1_/*T*_3_)*E*^*∗*^, *T*_1_≜*μ*+*k*_1_+*ε*, *T*_2_≜*μ*+*ϑ*+*γ*, and *T*_3_≜*μ*+*ϑ*+*k*_2_, *θ*≜*m*+*μ*.

**Proof**

The equilibrium point satisfies the following system of equations:

(14) $$\begin{array}{c} \left\{\begin{array}{c} -\beta IS+\Lambda \left(1-m\right)+k_{2}W-mS-\mu S=0,\\ \beta IS-k_{1}E-\varepsilon E-\mu E=0,\\ k_{1}E-\vartheta W-k_{2}W-\mu W=0,\\ \varepsilon E-\gamma I-\vartheta I-\mu I=0. \end{array}\right. \end{array}$$

Noticing that if *I*=0, we can obtain *P*_0_(0,0, *S*_0_, 0).

If *I* ≠ 0, as a result of the third and fourth equations of (14), we have

(15) $$\begin{array}{c} I^{*}=\frac{\varepsilon }{T_{2}}E^{*},\\ W^{*}=\frac{k_{1}}{T_{3}}E^{*}. \end{array}$$

Substituting *I*^*∗*^ and *W*^*∗*^ in the first and second equations of (14), we conclude that

(16) $$\begin{array}{c} S^{*}=\frac{T_{1}T_{2}}{\beta \varepsilon },\\ E^{*}=\frac{T_{3}\left[T_{1}T_{2}\theta -\beta \varepsilon \Lambda \left(1-m\right)\right]}{\beta \varepsilon \left(k_{1}k_{2}-T_{1}T_{3}\right)},\\ =\frac{T_{3}T_{1}T_{2}\theta \left(1-R_{0}\right)}{\beta \varepsilon \left(k_{1}k_{2}-T_{1}T_{3}\right)}, \end{array}$$

where *T*_1_≜*μ*+*k*_1_+*ε*, *T*_2_≜*μ*+*ϑ*+*γ*, and *T*_3_≜*μ*+*ϑ*+*k*_2_, *θ*≜*m*+*μ*.Thanks to

(17) $$\begin{array}{c} k_{1}k_{2}-T_{1}T_{3}=k_{1}k_{2}-\left(\mu +k_{1}+\varepsilon \right)\left(\mu +\vartheta +k_{2}\right)\\ =-\left(\mu +\varepsilon \right)\left(\mu +\vartheta \right)-k_{1}\left(\mu +\vartheta \right)-k_{2}\left(\mu +\varepsilon \right)<0. \end{array}$$

Suppose that *R*_0_ > 1; obviously, there is *E*^*∗*^ > 0. Then, in this case, it follows that *P*^*∗*^(*E*^*∗*^, *I*^*∗*^, *S*^*∗*^, *W*^*∗*^). Otherwise, there would be no *P*^*∗*^.

## 4. Stability of Equilibrium Points

It is worth noting that the existence and unique conditions of equilibrium points have been proved in Theorem 1. Next, we will focus on the stability of model (2) with respect to the equilibrium points in this section.

**Theorem 2 .**

If *R*_0_ < 1, then *P*_0_(0,0, *S*_0_, 0) of model (2) is locally asymptotically stable in Ω.

**Proof**

We linearize system (2) around *P*_0_(0,0, *S*_0_, 0). The matrix of the linearization at *P*_0_(0,0, *S*_0_, 0) is given by

(18) $$\begin{array}{c} J\left(P_{0}\right)=\left(\begin{array}{cccc} -T_{1} & \beta S_{0} & 0 & 0\\ \varepsilon & -T_{2} & 0 & 0\\ 0 & -\beta S_{0} & -\theta & k_{2}\\ k_{1} & 0 & 0 & -T_{3} \end{array}\right), \end{array}$$

where *T*_1_=*μ*+*k*_1_+*ε*, *T*_2_=*μ*+*ϑ*+*γ*, *T*_3_=*μ*+*ϑ*+*k*_2_, and *θ*=*m*+*μ*.

The formula of characteristic equation for **J**(*P*_0_) being

(19) $$\begin{array}{c} f\left(\lambda \right)=\left(\lambda +T_{1}\right)\left(\lambda +T_{2}\right)\left(\lambda +T_{3}\right)\left(\lambda +\theta \right)-\beta S_{0}\varepsilon \left(\lambda +\theta \right)\left(\lambda +T_{3}\right)=0, \end{array}$$

which leads to

(20) $$\begin{array}{c} \left(\lambda +\theta \right)\left(\lambda +T_{3}\right)\left[\left(\lambda +T_{1}\right)\left(\lambda +T_{2}\right)-\beta S_{0}\varepsilon \right]=0. \end{array}$$

Clearly, (20) always has negative roots *λ*_1_=−*θ* and *λ*_2_=−*T*_3_. All other roots are determined by

(21) $$\begin{array}{c} \left(\lambda +T_{1}\right)\left(\lambda +T_{2}\right)-\beta \varepsilon S_{0}=0. \end{array}$$

Substituting (13) into (21) yields

(22) $$\begin{array}{c} \left(\lambda +T_{1}\right)\left(\lambda +T_{2}\right)-T_{1}T_{2}R_{0}=0, \end{array}$$

which is of the form *λ*^2^+*b*_1_*λ*+*b*_2_=0, where *b*_1_=*T*_1_+*T*_2_ and *b*_2_=*T*_1_*T*_2_(1 − *R*_0_).

When *R*_0_ < 1, we conclude that Φ_1_=*b*_1_=*T*_1_+*T*_2_ > 0 and Φ_2_=*b*_1_*b*_2_=*T*_1_*T*_2_(*T*_1_+*T*_2_)(1 − *R*_0_) > 0. According to Lemma 1 [14], there exist negative real parts for all roots of (21). Therefore, *P*_0_(0,0, *S*_0_, 0) of (2) is locally asymptotically stable.

**Theorem 3 .**

If *R*_0_ > 1, *P*^*∗*^(*E*^*∗*^, *I*^*∗*^, *S*^*∗*^, *W*^*∗*^) is locally asymptotically stable in Ω^0^.

**Proof**

From Theorem 1, there exists *P*^*∗*^ in model (2) only if *R*_0_ > 1.Then, the Jacobian matrix of model (2) at *P*^*∗*^(*E*^*∗*^, *I*^*∗*^, *S*^*∗*^, *W*^*∗*^) is presented as follows

(23) $$\begin{array}{c} J\left(P^{*}\right)=\left(\begin{array}{cccc} -T_{1} & \beta S^{*} & \beta I^{*} & 0\\ \varepsilon & -T_{2} & 0 & 0\\ 0 & -\beta S^{*} & -\beta I^{*}-\theta & k_{2}\\ k_{1} & 0 & 0 & -T_{3} \end{array}\right), \end{array}$$

where *T*_1_=*μ*+*k*_1_+*ε*, *T*_2_=*μ*+*γ*+*ϑ*, *T*_3_=*μ*+*ϑ*+*k*_2_, and *θ*=*m*+*μ*.

The characteristic equation of **J**(*P*^*∗*^) is

(24) $$\begin{array}{c} g\left(\lambda \right)=\left(\lambda +T_{1}\right)\left(\lambda +T_{2}\right)\left(\lambda +T_{3}\right)\left(\lambda +\beta I^{*}+\theta \right)-\beta \varepsilon S^{*}\left(\lambda +T_{3}\right)\left(\lambda +\theta \right)-k_{1}k_{2}\beta I^{*}\left(\lambda +T_{2}\right)=0, \end{array}$$

that is,

(25) $$\begin{array}{c} \lambda^{4}+b_{1}\lambda^{3}+b_{2}\lambda^{2}+b_{3}\lambda +b_{4}=0, \end{array}$$

where

(26) $$\begin{array}{c} b_{1}=T_{1}+T_{2}+T_{3}+\beta I^{*}+\theta >0,\\ b_{2}=T_{1}T_{3}+T_{2}T_{3}+\left(\beta I^{*}+\theta \right)\left(T_{1}+T_{2}+T_{3}\right)>0,\\ b_{3}=\beta I^{*}\left(T_{1}T_{2}+T_{2}T_{3}\right)+\theta \left(T_{1}T_{3}+T_{2}T_{3}\right)+\beta I^{*}\left(T_{1}T_{3}-k_{1}k_{2}\right),\\ b_{4}=\beta I^{*}T_{2}\left(T_{1}T_{3}-k_{1}k_{2}\right). \end{array}$$

Considering that *T*_1_*T*_3_ − *k*_1_*k*_2_=(*μ*+*k*_1_+*ε*)(*μ*+*ϑ*+*k*_2_) − *k*_1_*k*_2_ > 0, we arrive at *b*_3_ > 0, *b*_4_ > 0.

Owing to

(27) $$\begin{array}{c} \Phi_{1}=b_{1}=T_{1}+T_{2}+T_{3}+\beta I^{*}+\theta >0,\\ \Phi_{2}=b_{1}b_{2}-b_{3}\\ =\left(T_{1}+T_{2}+T_{3}+\beta I^{*}+\theta \right)\left[T_{1}T_{3}+T_{2}T_{3}+\left(\beta I^{*}+\theta \right)\left(T_{1}+T_{2}+T_{3}\right)\right]\\ -\left[\beta I^{*}\left(T_{1}T_{2}+T_{2}T_{3}\right)+\theta \left(T_{1}T_{3}+T_{2}T_{3}\right)+\beta I^{*}\left(T_{1}T_{3}-k_{1}k_{2}\right)\right]\\ =\left(T_{1}+T_{2}+T_{3}\right)\left[\left(T_{1}+T_{2}+T_{3}+\beta I^{*}+\theta \right)\left(\beta I^{*}+\theta \right)+\left(T_{1}T_{3}+T_{2}T_{3}\right)\right]\\ +\beta I^{*}k_{1}k_{2}-\beta I^{*}T_{1}T_{2}>0,\\ \Phi_{3}=b_{3}\left(b_{1}b_{2}-b_{3}\right)-b_{1}{}^{2}b_{4}=b_{3}\Phi_{2}-b_{1}{}^{2}b_{4}\\ =\left[\beta I^{*}\left(T_{1}T_{2}+T_{2}T_{3}\right)+\theta \left(T_{1}T_{3}+T_{2}T_{3}\right)+\beta I^{*}\left(T_{1}T_{3}-k_{1}k_{2}\right)\right]\\ \left\{\left(T_{1}+T_{2}+T_{3}\right)\left[\left(T_{1}+T_{2}+T_{3}+\beta I^{*}+\theta \right)\left(\beta I^{*}+\theta \right)+\left(T_{1}T_{3}+T_{2}T_{3}\right)\right]+\beta I^{*}\left(k_{1}k_{2}-T_{1}T_{2}\right)\right\}\\ -{\left(T_{1}+T_{2}+T_{3}+\beta I^{*}+\theta \right)}^{2}\left[\beta I^{*}T_{2}\left(T_{1}T_{3}-k_{1}k_{2}\right)\right]\\ =\beta I^{*}{\left(\beta I^{*}+\theta \right)}^{2}\left(T_{1}T_{3}-k_{1}k_{2}\right)\left(T_{1}+T_{3}\right)\\ +\beta I^{*}\left(\beta I^{*}+\theta \right)\left(T_{1}+T_{2}+T_{3}\right)\left[\left(T_{1}T_{2}+T_{2}T_{3}\right)\left(T_{1}+T_{2}+T_{3}\right)+T_{2}k_{1}k_{2}-T_{1}T_{2}T_{3}\right]\\ +\beta I^{*}\left(T_{1}+T_{2}+T_{3}\right){\left(T_{2}T_{3}\right)}^{2}+\Phi_{2}\left[\beta I^{*}\left(k_{1}k_{2}-T_{1}T_{3}\right)+\theta \left(T_{1}T_{3}+T_{2}T_{3}\right)\right]>0,\\ \Phi_{4}=b_{4}\Phi_{3}=\beta I^{*}T_{2}\left(T_{1}T_{3}-k_{1}k_{2}\right)\Phi_{3}>0. \end{array}$$

It follows from Lemma 1 [14] that there exist negative real parts for all roots of (24). Therefore, *P*^*∗*^(*E*^*∗*^, *I*^*∗*^, *S*^*∗*^, *W*^*∗*^) is locally asymptotically stable. The corresponding global asymptotic stability will be verified in the numerical simulation.

**Theorem 4 .**

If *R*_0_ < 1, *P*_0_(0,0, *S*_0_, 0) of model (2) is globally asymptotically stable in Ω.

**Proof**

Define the following Lyapunov function as

(28) $$\begin{array}{c} ℒ\left(t\right)=\varepsilon E\left(t\right)+\left(\mu +k_{1}+\varepsilon \right)I\left(t\right). \end{array}$$

Obviously, we have ℒ(*t*) ≥ 0. Furthermore, ℒ(*t*)=0 if and only if both *E*(*t*)=0 and *I*(*t*)=0.

The derivative of ℒ(*t*) along model (2) is

(29) $$\begin{array}{c} \frac{\text{d}ℒ\left(t\right)}{\text{d}t}|\left(4\right)=\varepsilon \left(\beta I\left(t\right)S\left(t\right)-\mu E\left(t\right)-k_{1}E\left(t\right)-\varepsilon E\left(t\right)\right)+\left(\mu +k_{1}+\varepsilon \right)\left(\varepsilon E\left(t\right)-\mu I\left(t\right)-\gamma I\left(t\right)-\vartheta I\left(t\right)\right),\\ =\beta \varepsilon I\left(t\right)S\left(t\right)-\left(\mu +k_{1}+\varepsilon \right)\left(\mu +\gamma +\vartheta \right)I\left(t\right),\\ =I\left(t\right)\left[\beta \varepsilon S\left(t\right)-\left(\mu +k_{1}+\varepsilon \right)\left(\mu +\gamma +\vartheta \right)\right]\\ \leq I\left(t\right)\left[\beta \varepsilon S_{0}-\left(\mu +k_{1}+\varepsilon \right)\left(\mu +\gamma +\vartheta \right)\right]\\ =I\left(t\right)\left(\mu +k_{1}+\varepsilon \right)\left(\mu +\gamma +\vartheta \right)\left(R_{0}-1\right). \end{array}$$

When *R*_0_ < 1, we have dℒ(*t*)/d*t* ≤ 0. Furthermore, we obtain dℒ(*t*)/d*t*=0 if and only if *I*(*t*)=0. Consequently, the largest set of compact invariants in {(*S*, *E*, *W*, *I*)*|d*ℒ(*t*)/d*t*=0} is the single point set {*P*_0_} when *R*_0_ < 1. With the aid of Lemma 2 [15] and Lemma 3 [16], *P*_0_(0,0, *S*_0_, 0) of (2) is globally asymptotically stable in Ω when *R*_0_ < 1.

## 5. Model Simulations

In the section, first the relevant results in Section 4 will be verified. Subsequently, the impact of vaccination and government control on infectious diseases will be analyzed. Parameters are listed in Table 1.

The initial values for (*S* (0), *E* (0), *I* (0), *R* (0)) is set as (120, 0, 15, 1, 0), (70, 0, 15, 1, 50), and (20, 0, 15, 1, 100). *m* and *k*_1_ are variables, and the other parameters are set to constant values in Table 1.

In Case 1, we set *m*=0.8 and *k*_1_=0.6. Then, *R*_0_=0.9802 < 1 and *P*_0_(0,0, *S*_0_, 0)=(0,0,3.4091, 0). Then, we simulate the changes in the number of these four populations under the condition of *R*_0_ < 1. In Case 2, we set *m*=0.35 and *k*_1_=0.3. Then, *R*_0_=8.1769 > 1 and *P*^*∗*^(*E*^*∗*^, *I*^*∗*^, *S*^*∗*^, *W*^*∗*^)=(7.2730, 6.1898, 2.7730, 2.4516). Similarly, the population size for the condition *R*_0_ > 1 is simulated as well. The relative results are illustrated in Figure 2. The first row shows the changes in population size for different initial settings in case 1, and the second row shows the changes in population size for case 2.

From Figure 2, it can be concluded that the decrease in the initial value of susceptible individuals at the beginning of the outbreak leads to a shorter duration of the epidemic. Meanwhile, the peak of confirmed cases reaches a lower level in almost unanimous time.

Focusing on Figures 2(a) and 2(d), it is evident that the equilibria of (2) are globally asymptotically stable. Correspondingly, three conclusions can be drawn: (1) compared to Case 1, the amount of the four populations in Case 2 starts to stabilize after about day 160, however, about 20 days later than in Case 1. (2) In Case 2, neither the exposed nor the infected populations can achieve disappearance, i.e., the epidemic will persist. However, as illustrated in Case 1, once the four populations have stabilized, the total population will consist entirely of the susceptible and recovered population that has been immunized. This is a high-priority objective for epidemic control. (3) The exposed and infected populations in Case 2 consume a similar amount of time as in Case 1, but reach a higher peak. Hence, we can infer from these findings that government involvement and vaccination both have an impact on the epidemic dynamics.

From the analysis above, we can obtain that *m* as well as *k*_1_ has a beneficial effect on the prevention and control of the epidemic. Consequently, we will specifically investigate the effectiveness of *m* and *k*_1_ for the control of COVID-19. The initial value is set as (120, 0, 15, 1, 0). Changes in the amount of quarantined virus exposed population *W*(*t*) and infected population *I*(*t*) will be observed.

In Case 3, we set *m* = 0.35 and *k*_1_ = 0.6 initially. And, the basic reproduction number *R*_0_=6.5149 > 1. From Figure 3(a), we find the blue parts of the *W*(*t*) and *I*(*t*) curves converge quickly after about day 150 and reach dynamic equilibrium, in which case extinction of the epidemic disease cannot be achieved. On day 220, we raise *m* to *m* = 0.8, at which point *R*_0_=0.9802 < 1. Obviously, *I*(*t*) and *W*(*t*) both started to decline rapidly from day 220 and dropped below 1 around day 260. Hence, it can be concluded that the increase of vaccination success rate *m* has a strong and efficient effect on the implementation of the COVID-19 control efforts.

In Case 4, we set *m* = 0.35 and *k*_1_ = 0.2 initially, i.e., reduce the government control rate *k*_1_ on the basis of case 3 at the stage when no epidemic control work is carried out. Subsequently, both *m* and *k*_1_ were increased to be consistent with the parameter values on day 220 in Case 3. Thus, Figure 3(b) can be obtained. Comparison Figures 3(a) and 3(b), it can be found that, with a higher the initial *k*_1_, the peak number of *W*(*t*) will rise by about 93.5%, but the peak number of *I*(*t*) will drop by about 17.7%. When the epidemic control work begins on day 220, the number of *W*(t) exhibits an increasing trend followed by a declining trend, which would result in higher epidemic control costs compared to that of Case 3.

By calculating the time points of no new *W*(*t*) and *I*(*t*) addition after the control work, the results of day 258 and day 261 of Case 3 can be obtained, respectively. Meanwhile, we can obtain the results of day 264 and day 269 of Case 4. Consequently, if the implementation of the government's control work intensity can reach a high level in the early stage of the outbreak of COVID-19, it will help to shorten the time of control work with a reduction in new infection cases.

In Cases 3 and 4, we first simulate the process of epidemic from an outbreak to a convergence to equilibrium without extinction. Then, we insert control means immediately afterwards including vaccination and government intervention which make the epidemic go to extinction, thus achieving the purpose of control. Next, we will investigate the role of *m* and *k*_1_ for epidemic control individually.

In Case 5, we fix *k*_1_ = *0.8* and adjust *m* under the condition of ensuring *R*_0_ < 1, so as to monitor variations in the number of *I*(*t*). Then, Figure 4(a) can be obtained. Under the limited condition of *R*_0_ < 1, we can determine that the three time points when the number of *I*(*t*) peaks all fell within the range of day 50 to day 100.

In Case 6, similarly, we fix *m* *=* *0.8* and adjust *k*_1_ to obtain Figure 4(b). From Figure 4(b), we can conclude that, with the improvement of *k*_1_, the time points when the three curves reach their peaks tend to be earlier. In other words, when *m* reaches a high level, the increase of *k*_1_ will simultaneously lead to two positive effects: an earlier point of time at which the number of *I*(*t*) peaks and peaks decline.

At the same time, we find, to *m* and *k*_1_, the corresponding sensitivity of *R*_0_ are not identical. Then, according to (4) in Section 3, the relationship between these two factors and *R*_0_ can be obtained, as shown in Figure 5. It can be obtained that *R*_0_ is more sensitive to *m*. Then, when *k*_1_ and *m* are, respectively, increased within the same numerical range, *m* has a greater benefit for the mitigation of the epidemic.

According to the simulation results obtained with, we find, the expansion of vaccination coverage, as well as the increase in government intervention contribute to the extinction of infectious diseases. Under the condition that *R*_0_ < 1, once there exists an increase in *m* and *k*_1_, it will bring a positive effect of reducing the number of confirmed cases. And, if government intervention continues to expand in the face of vaccination for universal access, an added effect of an earlier demise of the epidemic will be gained.

## 6. Conclusion and Strategies

In the present work, a SEWIR epidemic model with vaccination and government control is presented. The basic regeneration number *R*_0_ is calculated as the threshold which describes the extinction or persistence of the disease. By constructing the Lyapunov function and numerical simulations, it can be demonstrated that the disease-free equilibrium point of model (2) is globally asymptotically stable when *R*_0_ < 1 and the infectious disease will tend to die out over time; when *R*_0_ > 1, the endemic equilibrium point of model (2) is also globally asymptotically stable but will not achieve extinction but maintain dynamic equilibrium. In parallel, through extensive simulation experiments, we further study the impact of vaccination success and government control rates on the dynamics of the COVID-19 epidemic. In Case 3, we simulate the effect of vaccination on epidemic control. When only the vaccination success rate is adjusted from 0.35 to 0.8 and the government control rate is kept constant, the basic regeneration number *R*_0_ is reduced from 6.5194 to 0.9802, and the epidemic tends to extinction in about 40 days. Hence, we can obtain the first control strategy: advancing the progress of vaccine development for COVID-19 and improving the immunization success rate of the vaccine. In Case 4, we adjust both the vaccination success rate from 0.35 to 0.8 and the government control rate from 0.2 to 0.6. Compared to Case 3, the number of quarantined exposed population experiences an increase and then a decrease. For both cases, we can conclude that if the government double the rate of control in the early stage of the outbreak, the number of quarantined exposed population will increase by 93.5%, but the number of infected population will decrease by 17.7% successively. Therefore, a second control strategy can be obtained: promoting the progress of governmental efforts to contain the epidemic during its early stage: for example, to increase the frequency and scope of medical testing, to expand the investigation of people who have been in contact with positive patients, and to implement home quarantine for all people in certain region. Both of these strategies have good effect on the control of the epidemic.

The results above suggest that improving the immunization success rate of vaccine, enhancing vaccination efforts and government intervention can be used as strategies to control the epidemic during COIVD-19. However, the huge impact of a long-term region-wide quarantine on the daily life of public and the enormous consumption of human and material resources during the quarantine cannot be ignored. Consequently, it can only be used as a short-term expedient measure. In order to fundamentally eliminate the epidemic, it is necessary to vigorously promote vaccination and improve the quality of vaccines to reduce the diagnosis rate and mortality rate.

Nevertheless, these results must be interpreted with caution, and there are several limitations that cannot be ignored. First, cultural differences and social factors between countries were not taken into account in the modeling process. Large-scale and long-term medical isolation measures are not applicable to all countries. Second, economic factors were also not considered. The proposed optimal prevention and control strategy is relatively idealistic and has some implementation limitations. In subsequent studies, it will be considered again from this aspect as well as the perspective of vaccination methods and vaccination coverage.

## Figures and Tables

**Figure 1:** The transmission mechanism figure of the VGC-SEWIR model.

**Figure 2:** Equilibria global asymptotic stability of model (2). The first row is the case 1, and the second row is the case 2. (a, d) Initial values set as (120, 0, 15, 1, 0); (b, e) initial values set as (70, 0, 15, 1, 50); (c, f) initial values set as (20, 0, 15, 1, 100). (a) Case 1: initial value (120, 0, 15, 1, 0). (b) Case 1: initial value (70, 0, 15, 1, 50). (c) Case 1: initial value (20, 0, 15, 1, 100). (d) Case 2: initial values (120, 0, 15, 1, 0). (e) Case 2: initial values set as (70, 0, 15, 1, 50). (f) Case 2: initial values set as (20, 0, 15, 1, 100).

**Figure 3:** Effect of parameters *m* and *k*_1_ on quarantined virus exposed population and infected population. (a) Case 3: adjustment of parameter *m* only. (b) Case 4: simultaneous adjustment of parameters *m* and *k*_1_.

**Figure 4:** Sensitivity analysis of parameter *m* and *k*_1_ to infected population when *R*_*0*_ < 1. (a) Case 5: sensitivity of parameter *m*. (b) Case 6: sensitivity of parameter *m* and *k*_1_.

**Figure 5:** The relationship between parameter *m* and *k*_1_ on the basic regeneration number *R*_0_.

**Table 1:** Parameters definition and estimated values.

Parameters	Definition	Value
Λ	Population replenishment rate	15
*β*	Infected population level infection rate	0.5
*μ*	Natural mortality rate	0.08
*ε*	Conversion from unquarantined virus exposed population to infected populations	0.8
*γ*	Disease mortality	0.06
*m*	Vaccination success rate	Variable
*k*_1_	Government control rate	Variable
*ϑ*	Recovery rate	0.8
*k*_2_	Autoviral immunity rate	0.01

## Data Availability

The dataset used to support the findings of this study are available from the corresponding author upon request.
